# Resiliency Assessment of Power Systems Using Deep Reinforcement Learning

**DOI:** 10.1155/2022/2017366

**Published:** 2022-04-07

**Authors:** Mariam Ibrahim, Ahmad Alsheikh, Ruba Elhafiz

**Affiliations:** ^1^Department of Mechatronics Engineering, German Jordanian University, Amman 11180, Jordan; ^2^Department of Natural Science & Industrial Engineering, Deggendorf Institute of Technology, Deggendorf 94469, Germany

## Abstract

Evaluating the resiliency of power systems against abnormal operational conditions is crucial for adapting effective actions in planning and operation. This paper introduces the level-of-resilience (LoR) measure to assess power system resiliency in terms of the minimum number of faults needed to produce a system outage (blackout) under sequential topology attacks. Four deep reinforcement learning (DRL)-based agents: deep *Q*-network (DQN), double DQN, the REINFORCE (Monte-Carlo policy gradient), and REINFORCE with baseline are used to determine the LoR. In this paper, three case studies based on IEEE 6-bus test system are investigated. The results demonstrate that the double DQN network agent achieved the highest success rate, and it was the fastest among the other agents. Thus, it can be an efficient agent for resiliency evaluation.

## 1. Introduction

The deployment of recent technologies in communication, computing, and control of smart grids can be suitable for clients and electrical facilities. Energy infrastructures are natively connected to other areas of demanding infrastructures, and their supply breaking can have disastrous cascading results [1]. One of the important features that is essential in today's smart grids is to run resiliently when attacks/faults and other contingencies occur.

Determining the resilience of power systems (PSs) has been a subject of concern in latest years. Stochastic and statistical analysis techniques are used to evaluate power system resilience [2]. While these techniques can aid understanding the system resilience to large-scale contingencies, however, they are not always appropriate when evaluating resilience in the presence of malicious sources. These methods are based on the comparably simple DC model, which does not consider effects like voltage breakdown that may happen during a cascade. Also, there is a need to enhance their data, sampling ways, and the extent of models and effects represented [3]. Accordingly, it is essential to investigate new approaches to evaluate the resilience of the grid using the more realistic and scalable AC models.

The applications of machine learning (ML) algorithms are identified by Olowononi et al. [4] in the field of security and resiliency of the power grid. Their target is to effectively survey the interactions among resilient grid using ML and resilient ML when used in the grid. The power system's cybersecurity and ML have a wide range of interdisciplinary crossways between them. For instance, reinforcement and deep learning (DL) can be used to build smart models for applying malware classification, observing the use of the intrusion detection and prevention systems (IDS/IPS), and implementing threat intelligence sensing [5].

Reinforcement learning (RL) is one of the established ML approaches [6]. RL does not depend directly on data sets but has an agent that is placed in an anonymous environment and can receive feedbacks in form of rewards by making actions that can result in maximizing cumulative rewards, so the agent learns from its own experience. The agent focuses on finding an optimal policy rather than analyzing data as compared to supervised and unsupervised learning. The environment usually has dynamics that are unknown to the agent.

The DL approaches grant computational models that are created of numerous processing layers to learn representations of data with various levels of abstraction. These approaches have effectively enhanced the visual object recognition, speech recognition, and numerous realms [7]. The combination of RL with DL techniques (DRL) is most useful in problems with a high dimensional state-space which makes it suitable for evaluating the resilience of power systems. Classical RL techniques has a complex design issue in the decision of features. Nonetheless, DRL has been rewarding in difficult assignments with a lower prior knowledge [8]. The recent advancement in DL techniques is summarized by Dick et al. [1] for creating machine vision models. The current applications of this technology are also investigated to improve the resiliency of critical infrastructure protection (CIP).

Several works investigated the cybersecurity of power grids using RL and DRL. For instance, Dibaji et al. [9] considered cyber physical systems' security from systems and control perspectives in general, and shortly discussed the possibilities of using RL and DRL to this purpose. *Q*-learning was proposed by Yan et al. [10] to interpret the transmission grid vulnerability against sequential topology attacks and determine critical attack sequences taking into account physical system behaviors. A modified *Q*-learning (termed the nearest sequence memory *Q*-learning) was adopted by Wang et al. [11] to evaluate threats imposed by false data injection attack on voltage control of a power system. Test results revealed that even if a few substations are attacked, a voltage collapse with its consequences can happen in the system.

Secure state estimation using multiagent reinforcement learning was dealt by He et al. [12] with the assumption that measurements are sent over a wireless network under jamming attacks. The antijamming game framework was used to determine the optimal path against an intelligent attacker. He et al. [13] considered secure-state estimation with risk-averse transmission path selection method that is based on RL concept. They demonstrated how the proposed approach can improve secure-state estimation robustness.

The use of RL was discussed by Oozeer et al. [14] in a general framework of cognitive risk control for cyber-attacks in smart grids. RL was presented by Chen et al. [15] to evaluate false data injection attacks against automatic voltage control of power systems (in normal operating states). A *Q*-learning algorithm with the nearest sequence memory was employed for online learning of attacking strategy. The optimal attack strategy was modelled as a partially observable Markov decision process. Based on kernel density estimation, a bad data detection and correction technique was presented to reduce the disruptive influence of the attacks.  Table 1 shows some recent studies that were performed on smart grid system security using RL and DRL.

The novelty of this work lies in evaluating power system's resiliency level (LoR) under sequential topological attacks/faults using DRL techniques. The framework design methodology is based on using four DRL agents which are trained and optimized with the aim of determining the minimum number of faults required to black out the system. This number is used to determine the LoR for three different topologies of IEEE 6-bus system case study under single and three-phase attack scenarios. The performance of the tested DRL agents was compared. The double DQN agent was stable and achieved the highest success rate among all agents. Thus, it can be used for resilience studies that investigate the system's ability to withstand attacks/faults by aiding system designers to select the most resilient system's topology. The rest of the paper is straightened out as follows: Section 2 illustrates power system's topologies along with the attack/faults scenarios.  Section 3 presents the resiliency measure formulation and the DRL techniques. Experimental results are shown in Section 4.  Section 5 summarizes and presents certain future directions.

### 1.1. Acronyms and Notations

Table 2 illustrates the acronyms and notations used through the paper.

## 2. Preliminaries

### 2.1. Electric Power Grid Topology

An electrical power grid is a complementary network for carrying electricity from producers to consumers. Electrical grids differ in size from serving whole countries through national grids to cross-continents through transnational grids [21]. Three power system topologies were considered in this paper. These are PS1, PS2, and PS3, respectively, as shown in Figures 1to 3. They have identical buses, generation, and load units. Each system is a three-phase electric power system that consists of three loads (each has an active power of 70 Mw), three generators (two photovoltaic (PV) generators and one swing) with active power of 50 Mw for each, six buses and 36 transmission lines. The power system PS1 is an IEEE 6-bus system introduced by Kennedy [22]. PS2 was generated by altering PS1's topology, while PS3 can be described as a fully connected system where all the RLC circuits are connected to each other.

In PS1, PS2, and PS3, the loads L1, L2, and L3 are connected to buses 4, 5, and 6, respectively. Nonetheless, the generators Swing, PV1, and PV2 are connected to buses 1, 2, and 3, respectively. The values of RLC of lines are also equal in all the three grids. The topology differences can be shown in the transmission line connections which resulted in altering the potential paths of current flow.

### 2.2. Faults Scenarios

Typically, a power system performs well under balanced conditions. However, the system might become unbalanced due to several reasons, such as natural disturbances (e.g., earthquakes, lightning, and high-speed winds), tree falling on the lines, and insulation failure. These reasons can lead to short-circuits or a fault in the lines [22]. The most harming faults in power systems are short-circuit faults because their occurrence can result into a significant increase in the electrical current. Nonetheless, there exists two types of short-circuit faults: symmetric and asymmetric [23].

In a symmetric fault, all the phases are short-circuited to each other and often to earth. Such a fault is balanced in the sense that the system remains symmetrical, or in other words, the lines are displaced by an equal angle. It is the most relentless type of faults, including the largest current. Yet, it rarely materializes [24], such as a three-phase line to the ground fault (L–L–L–G) where the fault occurs between the three phases and the ground of the system. The asymmetrical fault gives rise to asymmetrical current, that is, the current is differing in magnitude and phase in the three phases of the power system. When a short-circuit occurs, the current comes into its peak value rapidly, and then it reduces exponentially with time through three different states: subtransient, transient, and permanent states [25]. Examples of asymmetrical faults are single line-to-ground (L–G) fault, line-to-line fault (L–L), and double line-to-ground (L–L–G) fault. In this work, the asymmetric (L–L–G) and symmetric (L–L–L–G) faults were considered against the three topologies.

## 3. Resiliency Measure and DRL Techniques

### 3.1. Resiliency Measure Formulation

LoR is the factor that is employed to hold the evolution of system's features through the variations of system's modes of operation under a sequence of fault and recovery actions. For a number of PSs under a sequence of faults/attacks (an attack scenario), suppose the resulting system modes are represented by *Z*_*0*_*⟶Z*_*1*_*⟶…⟶Z*_*m*_, where *Z*_*0*_ is the initial mode, while *Z*_*h*_ is the mode after the *h*th fault and reconfiguration (*h* = 1,…, *m*). A power system is more resilient if it needed a larger number of faults/attacks *N* over all possible attack scenarios *M* before its outage. This factor can be determined by using a reinforcement agent who finds the optimal number of faults (by trial and failure) needed to produce a blackout. This is called an optimal policy.

**Definition 1 .**

Given a set of power systems with identical buses, generation, and load units, but with different topologies: PS ≡ ∪ PS_k_; *k*∈ {1,…, *y*}, where *y* is the number of the power systems, and a set of attack scenarios *M*, we say that the LoR(PS_i_) > LoR(PS-PS_i_) if:

*N*_*PSi*_ > *N*_*PS*−*PSi*_

### 3.2. DRL Algorithms

When the agent begins to learn, the agent will be in a state *S* of the environment, by selecting an action *A*, the agent can switch from one state to another. The transition probability between states, that is, *P*, denotes the probability of the state to which the agent will arrive to. When the agent conducts an action, the environment delivers a reward *R* as feedback. The model describes the reward function and transition probabilities. The agent's policy *π*(*S*) provides the strategy on which is the best/optimal action to be taken in a specific state with the aim of maximizing the cumulative rewards. Every state is identified with a value function *V*(*S*) predicting the expected number of future rewards that the agent will obtain in this state by choosing an optimal action under the current/other policy. The future reward (also called return) *G*_*t*_ is the total sum of discounted rewards in the future as represented by:

(1) $$\begin{array}{c} G_{t}=R_{t+1}+\gamma R_{t+2}+\cdots =\sum_{k=0}^{\infty }\gamma^{k}R_{t+k+1}, \end{array}$$

where *γ* ∈ [0, 1] is the discounting factor which penalizes the rewards in the future, so an agent can focus on the future reward rather than the immediate reward. Both policy and value functions are what the agent tries to learn in RL. The cooperation among the agent and the environment includes a sequence of actions and rewards evolving in time *t* = 1, 2,…, *T*, where *T* is time step at which the termination state is reached. During this process, the agent gathers information about the environment and gives decisions on which action to take next to precisely learn the best policy. The state, action, and reward at time step *t* can be represented as *S*_*t*_, *A*_*t*_, and *R*_*t*_, respectively. Therefore, the full cooperation sequence is represented by one episode (trajectory) and the sequence terminates at the terminal state: *S*_1_, *A*_1_, *R*_1_, *S*_2_, *A*_2_, *R*_2_,…, *S*_*T*_.

DQN was introduced by Mnih et al. [26] through a combination of *Q*-learning with a function approximator (neural network) to overcome the tabular limit of *Q*-learning. The algorithm was tested on Atari games and the agent was able to achieve the human level in Atari games. The inputs were raw pixels of the game so that the same agent can learn multiple games with no need for a special processing of the inputs. The past trials of combining *Q*-learning with function approximators in the past were not successful due to the deadly triad issue [27], where the model suffered from instability and divergence. This issue was solved by improving and stabilizing the training procedure of *Q*-learning using two methods of experience replay and periodically updated target. Here, DQN is a neural network model that receives states as inputs and produces action values *Q*(*S*; *θ*) for network parameters *θ*. The episode step *e*_*t*_=(*S*_*t*_, *A*_*t*_, *R*_*t*_, *S*_*t*+1_) is stored in one replay memory *D*_*t*_={*e*_1_,…, *e*_*t*_}, where *D*_*t*_ has experienced *e*_*t*_ tuples over many episodes. During *Q*-learning updates, samples are drawn randomly from the replay memory (called experience replay). Thus, one sample could be used many times. This was useful in reducing the correlation between samples, which resulted in a network that can learn without any overfitting. Moreover, the experience replay could reuse old experience, which resulted in a smooth learning and more efficient tuples samples.

In periodically updated target, DQN keeps a copy of the network with an identical architecture and initializes with the same parameters (weights values). The predicted *Q* from the target network will be used to update the main *Q*-network. The target network's parameters are not trained like the main network, instead they are periodically synchronized with the parameters of the main *Q*-network. The idea behind this is to serve the same goal as the experience buffer by reducing the correlation between samples using different parameters in the main *Q*-network with *θ* and *θ*^−^ for the target network. Thus, optimizing the *Q* values towards the target values. This has shown to stabilize the learning. Here, the target network with parameters *θ*^−^ is the same as the main *Q*-network except that its parameters are copied every C time steps. The C steps were chosen to be two steps so that *θ*_*t*_^−^ = *θ*_*t*_ and are kept fixed in all other steps. The main *Q*-network goal is to produce an estimation of the *Q* values for each action that can be taken from that state, but the objective is to find an optimal *Q* value that satisfy the Bellman optimality equation:

(2) $$\begin{array}{c} q_{*}\left(S,A\right)=Ε\left[R_{t+1}+\gamma \;{\text{max}}_{A^{\prime }}q_{*}\left(S^{\prime },A^{\prime }\right)\right]. \end{array}$$

For any state-action pair (*S*, *A*) at time *t*, the expected return from starting in state *S* selecting action *A* and following the optimal policy *q*_*∗*_ thereafter is going to be the expected reward we get from taking an action *A* in state *S*, which is *R*_*t*+1_ plus the maximum expected discounted return that can be achieved from any possible next state-action pair. Also, since the agent is following an optimal policy, the following state *S*′ will be the state from which the best possible next action *A*′ can be taken at time *t*+1 and the max_*A*′_*q*_*∗*_(*S*′, *A*′) is outputted from the target network. This will be used eventually to calculate the loss from the main *Q*-network which is calculated by comparing the generated *Q* values from the main *Q*-network to the target *Q* values from the right-hand side of the Bellman equation, where the objective here is to minimize this loss. After the loss is calculated, the parameters *θ* within the main *Q*-network are updated via Stochastic Gradient Descent (SGD) and backpropagation. This process is done repeatedly for each state in the environment until minimizing the loss and arriving to an approximate optimal *Q* value as follows:

(3) $$\begin{array}{c} \text{Loss}=q_{*}-q,\\ \text{Loss}=Ε\left[R_{t+1}+\gamma \;{\text{max}}_{A^{\prime }}q_{*}\left(S^{\prime },A^{\prime }\right)\right]-Ε\left[\overset{\infty }{\underset{k=0}{\sum }}\gamma^{k}R_{t+k+1}\right], \end{array}$$

which can be rewritten into the following equation:

(4) $$\begin{array}{c} \text{Loss}=y_{j}-Q\left({\text{S}}_{i},A_{i}|\theta \right),\\ y_{j}=R_{j}\;+\gamma \;{\text{max}}_{A^{\prime }}Q^{-}\left(S^{\prime },A^{\prime }|\theta^{-}\right). \end{array}$$

However, DQN has the drawback of overestimation in most cases. Normally, the overestimation is caused by *Q* value update rule of taking the maximum *Q* value of the new state. Therefore, a double DQN was proposed by Hado et al. [28] to overcome the overestimation of the DQN. Double DQN improved *Q* value update rule by selecting the action corresponding to the maximum *Q* value of the current *Q*-network rather than using the maximum *Q* value of the target *Q*-network.

To make sure that the selected action for the next state is the action with the highest value function (highest *Q* value), the current *Q* network is used to find the best action with the highest *Q* value (*A*_max_), then the target network is used to calculate the target *Q* value (*Q*^−^) of taking this action at the next state:

(5) $$\begin{array}{c} \text{Loss}=y_{j}-Q\left({\text{S}}_{i},A_{i}|\theta \right),\\ y_{j}=R_{j}+\gamma \;Q^{-}\left(S^{\prime },A_{\text{max}}|\theta^{-}\right), \end{array}$$

where

(6) $$\begin{array}{c} A_{\text{max}}={\text{arg max}}_{A^{\prime }}Q\left(\left(S^{\prime },A^{\prime }|\theta \right)\right). \end{array}$$

DQN and double DQN are concerned with learning a state-action value (*Q* value) function and then selecting actions based on this value, where the *Q* value indirectly evaluates the policy that the agent follows. On the other hand, policy gradient methods instead learn the policy *π* directly by a parameterized function *π*_*θ*_(*A|S*) with respect to  *θ*, where the objective function value relies on the policy. Thus, the algorithm goal is to optimize *θ* to determine the optimal value of the function *π*_*θ*_(*A|S*).

The REINFORCE [29] (Monte-Carlo policy gradient) is a model-free, online, on-policy reinforcement learning technique. REINFORCE depends on an estimated return by Monte-Carlo methods using episode samples to update the policy parameter *θ*. The policy gradient methods learn a policy function directly (instead of a *Q* function). On-policy, means that REINFORCE learns from trajectories generated by the current policy. The objective function for policy gradients is defined as follows:

(7) $$\begin{array}{c} J\left(\theta \right)=E\left[\overset{T-1}{\underset{t=1}{\sum }}R_{t+1}\right]. \end{array}$$

A useful way to learn an approximation policy is by directly maximizing the expected reward using a gradient method (i.e., policy gradient). It describes the gradient of the expected reward with respect to the parameters, where the objective function *J* is calculated to learn a policy that maximizes the cumulative future reward *R* to be received starting from any given time *t* until the terminal time *T*. The policy optimization process uses a gradient ascent with the partial derivative of the objective with respect to the policy parameter *θ* to maximize the objective function:

(8) $$\begin{array}{c} \theta \leftarrow \theta +\frac{\delta J\left(\theta \right)}{\delta \theta }. \end{array}$$

REINFORCE works because the expectation of the sample gradient is equal to the actual gradient as shown in the consecutive equation:

(9) $$\begin{array}{c} \nabla_{\theta }J\left(\theta \right)=E_{\pi }\left\{Q^{\pi }\left(s,a\right)\ln\;\pi_{\theta }\left(A|S\right)\right\},\\ =E_{\pi }\left[G_{t}\nabla_{\theta }\ln\;\pi_{\theta }\left(A_{t}|S_{t}\right)\right]. \end{array}$$

Here, one can measure  *G*_*t*_ from real sample full trajectories and employ it to update the policy gradient. A commonly used modification of REINFORCE is to subtract a baseline value from the return *G*_*t*_ to decrease the variance of gradient estimation, while keeping the bias unchanged. For example, a common baseline is to subtract state-value from action-value, and if adapted, one could use the advantage *δ*(*S*, *A*)=Q(S, A) − V(S) in the gradient ascent update. While training the agent for each training episode, the agent generates episode experience by following actor policy *μ*(*S*). The agent conducts actions until it arrives at the terminal state *S*_*T*_. The episode experience includes the sequence *S*_*1*_, *A*_1_, *R*_2_, *S*_2_,…, *S*_*T*−1_, *A*_*T*−1_, *R*_*T*_, *S*_*T*_. Then, the agent calculates the return *G*_*t*_ each time step. In case a baseline was used, then the advantage function *δ*_*t*_ is calculated employing the baseline value function estimated from the critic as given by:

(10) $$\begin{array}{c} \delta \left(s,a\right)=G_{t}-V\left(S_{t}|\theta_{v}\right). \end{array}$$

In fact, the REINFOR.

CE-with-baseline technique learns both a policy and a state-value function, but according to Sutton et al. [29], it will not be considered as an actor-critic method because the state-value function is used only as a baseline, not as a critic. This means that the critic will not be used for bootstrapping that illustrates updating the value estimate for a state from the estimated values of subsequent states. However, REINFORCE applies the state-value function only as a baseline for the state whose estimate is being updated. Afterwards, in reinforce with baseline, the agent accumulates the gradients for the actor network and critic network as represented by Wang et al. (11) and He et al. (12):

(11) $$\begin{array}{c} \text{d}\theta_{\mu }=\sum_{t=1}^{T-1}\delta_{t}\nabla_{\theta_{\mu }}\ln\;\mu \left({\text{S}}_{t}|\theta_{\mu }\right), \end{array}$$

(12) $$\begin{array}{c} d\theta_{v}=\sum_{t=1}^{T-1}\delta_{t}\nabla_{\theta_{v}}\text{V}\left({\text{S}}_{t}|\theta_{v}\right). \end{array}$$

Finally, the agent will update the actor parameter *θ*_*μ*_, and the state-value *θ*_*v*_ in case of a baseline, as shown by He et al. (13) and Oozeer and Haykin (14), respectively, where *α* and *β* are the learning rates.

(13) $$\begin{array}{c} \theta_{\mu }=\theta_{\mu }+\alpha \text{d}\theta_{\mu }, \end{array}$$

(14) $$\begin{array}{c} \theta_{v}=\theta_{v}+\beta \text{d}\theta_{v}. \end{array}$$

### 3.3. Agents Features

To train the agents, the topological line states were given as inputs (also called observations). The distribution of the faults for the three topologies PS1, PS2, and PS3 has resulted in 12 faults in L–L–L–G case and 36 faults for L–L–G case. Each fault is placed at each possible line where the current can flow through. Therefore, let  *I* = {1, 2,…, 12} and *K* = {1, 2,…, 36}. For every time step  *t*, an agent is given an observation  *s*_*t*_(*I*)={*s*_*t*_(1), *s*_*t*_(2),…, *s*_*t*_(12)} (for L–L – L–G case) or *s*_*t*_(*K*) = {*s*_*t*_(1), *s*_*t*_(2),…, *s*_*t*_(36)} (for L–L–G case). The initial state of each observation is *s*(*I*∨*K*) = 1 which means that the line is not faulted (in service), the current is available and can flow through the line. However, when a line is faulted (out of service), the line's state is switched to  *s*(*I*∨*K*) = 0, which means that the line is faulted, and the current cannot flow through this line as illustrated by:

(15) $$\begin{array}{c} s_{t}\left(I\vee K\right)=\left\{\begin{array}{cc} 1, & \text{if line}\left(I\vee K\right)\text{is in service at time }t,\\ 0, & \text{if line}\left(I\vee K\right)\text{is out of service at time }t. \end{array}\right) \end{array}$$

Likewise, in every time step *t*, the agent selects to defect one line out of the *I* or *K* possible faults, where *A*_*t*_ (*I*∨*K*)= 1. Once a fault is selected, the faulted line is disconnected, and the current is rerouted into other possible paths (if exists) toward loads. In addition, the reward function *R* is defined as follows:

(16) $$\begin{array}{c} R_{t+1}\left(S_{t},A_{t}\;\right)=\left\{\begin{array}{cc} -10, & \text{each }t\text{ step,}\\ -10, & \text{if }A_{t}\in We_{t},\\ 0, & \text{otherwise}. \end{array}\right) \end{array}$$

Each time step the agent selects a line to attack, the agent receives a negative reward. Therefore, the number of faults that is needed to cause an outage of the system equals to the time steps in this episode. Also, during an episode, the actions that are taken by the agent will be stored in a buffer *We*_*t*_ =(*A*_1_, *A*_2_,…, *A*_*T*−1_). The current action *A*_*t*_ taken by the agent at time *t* is compared to *We*_*t*_  to prevent the agent from repeating an action that was taken previously in the episode. By doing so, the agent can be trained with the aim of determining the minimum number of faults required to black out the system.

### 3.4. Networks Parameters

The DQN and double DQN agents were implemented by first defining the critic networks that get the observations as inputs. A critic network has two hidden layers each with 24 hidden neurons, and each hidden layer is connected with a rectified linear activation function (RELU) and passed to the output layer to find the *Q* value for each defined action. The optimizer for the critic network is ADAM, with a learning rate of 0.001. The gradient threshold parameter was set up and defined to be 1 to prevent any gradient explosion when the network back propagates to update the network weights. This usually happens when the gradients increase in magnitude exponentially, which results in an unstable training and can diverge within a few iterations. Gradient clipping can prevent gradient explosion by stabilizing the training at higher learning rates and in the presence of outliers. Gradient clipping enables networks to be trained faster and does not often affect the accuracy of the learned task [30].

Adding a regularization (L2 regularization factor) term for the weights to the loss function is one way to reduce overfitting [31]. Another parameter that is needed to train the agent is the experience buffer that is assigned with size of 3000 since the model is relatively small. The agent computes updates using a mini batch of experiences randomly sampled from the buffer with size of 64 which is large enough to reduce the variance when computing gradients, but it increases the computational effort. The discount factor that applies to future rewards during training is 0.9.

The REINFORCE agent is composed of an actor that has two hidden layers with 24 hidden neurons, and each hidden layer is connected with an RELU activation function. Likewise, the REINFORCE with baseline agent, was constructed of an actor and a baseline network. The baseline has two hidden layers with 24 hidden neurons with a RELU function. Similar to DQN agent, the gradient threshold was set to 1. Alongside an ADAM optimizer with a learning rate of 0.005 and a discount factor of 0.9, the learning rates for the two REINFORCE agents were optimized with different values until 0.005 was found to produce better results.

## 4. Experimental Results

The four agents were implemented using Simulink (Simscape Electrical) environment for the three topologies for the two cases of L–L–L–G and L–L–G fault scenarios, respectively. These agents are DQN, double DQN, REINFORCE, and REINFORCE with baseline. The results for the case of symmetrical L–L–L–G fault scenarios are shown in Figure 4.

The figure shows the training progress of the four agents, where it points out the success rate with the number of episodes. Each episode describes a scenario of lines outages the agent applies to cause a complete system blackout. It can be observed that the DQN agent successfully found a policy that is able to outage the three topologies with a high success rate. It shows also that the DQN agent learned faster than the other agents and was stable during the learning. The double DQN agent was slightly slower at the start of the training but later was stable and achieved a higher success rate than the DQN agent in the three topologies. However, the REINFORCE and the REINFORCE with baseline were slower in learning. The REINFORCE failed in the three topologies to converge and had lots of spikes, which explains that the agent was not stable during the training process. The REINFORCE with baseline succeeded to stabilize in PS3. But in PS1 and PS2, it was improving slowly, which means that by letting the agent train in more episodes, it will converge to an optimal policy. The agent cannot explore the action-state space efficiently. Thus, it takes longer time to find a good policy. It is worth mentioning that all the attempts to optimize the REINFORCE agent by adjusting the learning rate and the number of hidden neurons in the actor network were not sufficient to stabilize the learning procedure and to find an optimal sequence of actions.  Table 3 shows the minimum possible number of faults to outage the three systems PS1, PS2, and PS3, respectively, determined by the four agents. It can be shown that the double DQN was able to find a solution or a sequence of actions that results in system outage with a smaller number of faults as compared to the other agents in PS2.

Following Definition 1, the results illustrate that the third topology PS3 is the most resilient topology, as it needed 7 faults to black out the system. This is because PS3 has more redundant paths, so even if a line is faulted, the current can still flow through other paths towards the intended load.

For the second case of single-phase L–L–G fault scenarios, the results are illustrated in Figure 5. The results demonstrate that the double DQN network agent achieved a higher success rate, and it was faster than the other agents. Also, the agent was capable of finding the optimal number of faults for PS1, while the other agents could not find them. The results also illustrate that the REINFORCE agent failed once again to determine the optimal number of faults for the three topologies. Besides that, the agent was not stable, and the success rates were declining in PS1 and PS2, respectively. The REINFORCE with baseline was improving similar to symmetrical fault scenarios but needed longer training episodes to converge. The DQN agent had a similar behaviour to the double DQN agent but could not find the optimal number of faults in PS1.

Table 4 shows the minimum number of faults under single-phase L–L–G fault scenarios. It can be noted that the double DQN found a sequence of faults that was sufficient to outage PS1 with the minimum number of faults as compared to the other agents. The DQN, double DQN, and REINFORCE with baseline agents found the optimal solutions for PS2 and PS3, respectively. However, the REINFORCE agent could not find the solution for the three topologies. Following Definition 1, the results show that the third topology PS3 is the most resilient topology.

These results demonstrate that the double DQN agent is a powerful tool for resilience studies that investigate the system's ability to withstand attacks/faults. The double DQN was used to avoid the DQN's overestimation issue, by improving *Q* value updating rule when selecting the action corresponding to the maximum *Q* value of the current *Q*-network rather than using the maximum *Q* value of the target *Q*-network. In addition, the results illustrate for the REINFORCE agent how subtracting a baseline can help reduce the variance and stabilizing the agent. Yet, it needs more training episodes to converge.

## 5. Conclusion

A new measure for comparing the LoR was proposed for PSs) under attacks/faults. This measure is based on comparing the minimum number of faults that causes system outage by employing reinforcement learning approaches. The reinforcement learning agents were DQN, double DQN, the REINFORCE (Monte-Carlo policy gradient), and REINFORCE with baseline. The LoR of three different PS topologies under symmetrical and asymmetrical fault scenarios were compared. Experimental results showed that while the three PSs have the exact set of generators and have enclosed the same set of loads, yet, they had distinct resiliency levels due to their topological dissimilarity. The multipaths presented in PS3 topology supported the load's demands by the generation side. The results also showed that the double DQN agent was stable and achieved the highest success rate among all agents, as opposed to the REINFORCE agent that failed to determine the minimum number of faults for the three topologies under both symmetrical and asymmetrical faults. In this work, the agents were trained for a certain number of observations (current flow paths and lines availability states) and possible attacks/faults actions for three IEEE 6-bus topologies. However, investigating the LoR for other PSs topologies requires defining and training new agents properties with new observations and actions. As a future work, other factors need to be investigated like recovery time, stability, as well as checking the LoR of more topologies to determine the most resilient PS design. In addition to that further development on the resiliency enhancement can be obtained through the adaptation of DL and decision-making techniques.

## Figures and Tables

**Figure 1:** Power system PS1.

**Figure 2:** Power system PS2.

**Figure 3:** Power system PS3.

**Figure 4:** Results of DRL agents for the case of symmetrical L–L–L–G fault scenarios.

**Figure 5:** Results of DRL agents for the case of asymmetrical L–L–G fault scenarios.

**Table 1:** Recent studies on smart grid system security using RL and DRL.

Reference	System	Method	Attack	Recovery action	Aim	Limitations
[16]	Modified 9-bus system	Deep deterministic policy gradient (DDPG)	Multiswitch attacks and false data injection (FDI) attacks	Reclose the transmission lines lost in the cyber-attack by optimizing the reclosing time.	Reach the asynchrony in the power system by applying power blocking which will accelerate/decelerate the rotors of the generators	Owing to its continuous action space, it will not be suitable for topological resilience studies
[17]	IEEE 9, 14 and 30-bus systems	Deep *Q*-network (DQN)	Data integrity attacks	No recovery action	Evaluate the delay-alarm error rates, false-alarm error rates, and detect-failure rates for the systems	DQN suffers from overestimation
[18]	IEEE 30-bus system	Deep *Q*-network (DQN)	Coordinated cyber physical topology (CCPT) attacks	Control center can detect the line outage by using phasor measurement units (PMU) data	Investigate the coordinated topology attacks in smart grid which combine a physical topology attack and a cyber-topology attack	
[19]	Wood & Wollenberg 6-bus system and IEEE 30-bus system	*Q*-learning	Sequential attacks	Automatic generation control (AGC)	Identify the minimum number of attacks/actions to reach blackout threshold	*Q*-learning and SARSA techniques are limited to systems with small state-action space
[20]	IEEE 14-bus system	SARSA	False data injection (FDI), jamming, and denial of service (DoS) attacks	No recovery action	Formulation an online cyber-attack detection as a POMDP problem and propose a solution based on the model-free RL for POMDPs	
Our work	IEEE 6-bus system	Deep *Q*-network (DQN), double DQN, REINFORCE, and REINFORCE with baseline	Sequential attacks	Disconnecting the faulted transmission lines	Evaluating the resiliency of power systems against faults/attacks using DRL	Needs to investigate tabular methods such as *Q*-learning and SARSA to compare their performance with DRL methods

**Table 2:** Acronyms and notations used.

Category	Items/symbols	Description

Acronyms	LoR	Level-of-resilience
	PS	Power system
	DRL	Deep reinforcement learning
	DQN	Deep *Q*-network
	ML	Machine learning
	CIP	Critical infrastructure protection
	PV	Photovoltaic generator
	DDPG	Deep deterministic policy gradient
	FDA	False data injection
	*Q* value	State-action value
	(L–G)	Single line-to-ground fault
	(L–L)	Line-to-line fault
	(L–L–G)	Double line-to-ground

Notations	*π*(S)	Agent's policy
	V(S)	Value function
	R	Reward
	*G*_*t*_	Return
	*γ*	The discounting factor
	S	State
	A	Action
	*ϵ*	Probability of selecting an action
	*θ*, *θ*^−^	Weights
	*y*_*j*_	The value function target
	∇_*θ*_*J*(*θ*)	Gradient
	*π*_*θ*_(*A|S*)	Parameterized function with respect to *θ*
	*δ*(*S*, *A*)	The advantage function
	*μ*(S)	Actor policy
	*S*_*T*_	Terminal state
	*α*, *β*	The learning rates
	*Z*_*h*_	The mode after *h*th fault and reconfiguration
	*M*	A set of attack scenarios
	*N*	Number of faults/attacks

**Table 3:** Minimum number of faults under three-phase L–L–L–G fault scenarios.

PS/agent	DQN	Double DQN	REINFORCE	REINFORCE with baseline
**PS1**	6	6	6	6
**PS2**	6	5	6	6
**PS3**	7	7	7	7

**Table 4:** Minimum number of faults under single-phase L–L–G fault scenarios.

PS/agent	DQN	Double DQN	REINFORCE	REINFORCE with baseline
**PS1**	8	7	10	8
**PS2**	7	7	8	7
**PS3**	10	10	11	10

## Data Availability

The IEEE 6-Bus system load flow Simulink model was used from Mathworks (https://www.mathworks.com/matlabcentral/fileexchange/74690-ieee-6-bus-load-flow-simulink-model). It is provided free for academic research.

## References

[1] Dick K., Russell L., Souley Dosso Y., Kwamena F., Green J. R. (2019). Deep learning for critical infrastructure resilience. *Journal of Infrastructure Systems*.

[2] Bernstein A., Bienstock D., Hay D., Uzunoglu M., Zussman G. Power grid vulnerability to geographically correlated failures—analysis and control implications.

[3] Kelly-Gorham M. R., Hines P. D. H., Zhou K., Dobson I. (2020). Using utility outage statistics to quantify improvements in bulk power system resilience. *Electric Power Systems Research*.

[4] Olowononi F. O., Rawat D. B., Liu C. (2020). Resilient Machine Learning for Networked Cyber Physical Systems: A Survey for Machine Learning Security to Securing Machine Learning for Cps. *IEEE Communications Surveys & Tutorials*.

[5] Li J.-h. (2018). Cyber security meets artificial intelligence: a survey. *Frontiers of Information Technology & Electronic Engineering*.

[6] Russell S., Norvig P. (2002). *Artificial Intelligence: A Modern Approach*.

[7] LeCun Y., Bengio Y., Hinton G. (2015). Deep learning. *Nature*.

[8] François-Lavet V., Henderson P., Islam R., Bellemare M. G., Pineau J. (2018). An introduction to deep reinforcement learning. *Foundations and Trends in Machine Learning*.

[9] Dibaji S. M., Pirani M., Flamholz D. B., Annaswamy A. M., Johansson K. H., Chakrabortty A. (2019). A systems and control perspective of CPS security. *Annual Reviews in Control*.

[10] Yan J., He H., Zhong X., Tang Y. (2016). Q-learning-based Vulnerability Analysis of Smart Grid against Sequential Topology Attacks. *iEEE Transactions on Information Forensics and Security*.

[11] Wang Z., Chen Y., Liu F., Xia Y., Zhang X. (2018). Power System Security under False Data Injection Attacks with Exploitation and Exploration Based on Reinforcement Learning. *IEEE Access*.

[12] He J., Chen C., Zhu S., Yang B., Guan X. (2018). Antijamming game framework for secure state estimation in power systems. *IEEE Transactions on Industrial Informatics*.

[13] He J., Chen C., Zhu S., Yang B., Guan X. (2018). Risk-averse Transmission Path Selection for Secure State Estimation in Power Systems. *IEEE Internet of Things Journal*.

[14] Oozeer M. I., Haykin S. (2018). Cognitive Risk Control for Mitigating Cyber-Attack in Smart Grid. *IEEE Access*.

[15] Chen Y., Huang S., Liu F., Wang Z., Sun X. (2018). Evaluation of reinforcement learning-based false data injection attack to automatic voltage control. *IEEE Transactions on Smart Grid*.

[16] Wei F., Wan Z., He H. (2019). Cyber-attack recovery strategy for smart grid based on deep reinforcement learning. *IEEE Transactions on Smart Grid*.

[17] An D., Yang Q., Liu W., Zhang Y. (2019). Defending against data integrity attacks in smart grid: a deep reinforcement learning-based approach. *IEEE Access*.

[18] Wang Z., He H., Wan Z., Sun Y. (2020). Coordinated topology attacks in smart grid using deep reinforcement learning. *IEEE Transactions on Industrial Informatics*.

[19] Ni Z., Paul S., Zhong X., Wei Q. A reinforcement learning approach for sequential decision-making process of attacks in smart grid.

[20] Kurt M. N., Ogundijo O., Li C. (2018). Online cyber-attack detection in smart grid: a reinforcement learning approach. *IEEE Transactions on Smart Grid*.

[21] Negirla P., Druță R., Silea I. (2020). Availability improvements through data slicing in PLC smart grid networks. *Sensors*.

[22] Kennedy C. (2020). *IEEE 6 Bus Load Flow Simulink Model*.

[23] Afwah A., Mogadisho S., Osman E. D., Abdirahman A. (2017). *Three-Phase Fault Analysis on Transmission Line in MATLAB SIMULINK*.

[24] Paiva S., Coelho L. F. (2005). *Redes de Energia Eléctrica: uma análise sistémica*.

[25] Hewitson L., Brown M., Balakrishnan R. (2004). *Practical Power System protection*.

[26] Mnih V., Kavukcuoglu K., Silver D. (2015). Human-level control through deep reinforcement learning. *Nature*.

[27] Sutton R., Barto A. (2017). *Introduction to Reinforcement Learning*.

[28] Hado V. H., Guez A., Silver D. Deep reinforcement learning with double q-learning.

[29] Sutton R., David M. A., Satinder S. P., Yishay M. (1999). Policy gradient methods for reinforcement learning with function approximation. *News in Physiological Sciences*.

[30] Pascanu R., Mikolov T., Bengio Y. On the Difficulty of Training Recurrent Neural Networks.

[31] Murphy K. B. (2012). *Machine Learning: A Probabilistic Perspective*.

